The article "Early Diagnosis of Acute Ischemic Stroke by Brain Computed Tomography Perfusion Imaging Combined with Head and Neck Computed Tomography Angiography on Deep Learning Algorithm" was published in 2022. Journal: Contrast Media Mol Imaging.

# Early Diagnosis of Acute Ischemic Stroke by Brain Computed Tomography Perfusion Imaging Combined with Head and Neck Computed Tomography Angiography on Deep Learning Algorithm

**DOI:** 10.1155/2022/5373585

**Published:** 2022-05-09

**Authors:** Yi Yang, Jinjun Yang, Jiao Feng, Yi Wang

**Affiliations:** ^1^Department of Medical Imaging Centre, The First People's Hospital of Xianyang, Xianyang 712000, Shannxi, China; ^2^Department of Ultrasound Medicine, The First People's Hospital of Xianyang, Xianyang 712000, Shannxi, China

## Abstract

The purpose of the research was to discuss the application values of deep learning algorithm-based computed tomography perfusion (CTP) imaging combined with head and neck computed tomography angiography (CTA) in the diagnosis of ultra-early acute ischemic stroke. Firstly, 88 patients with acute ischemic stroke were selected as the research objects and performed with cerebral CTP and CTA examinations. In order to improve the effect of image diagnosis, a new deconvolution network model AD-CNNnet based on deep learning was proposed and used in patient CTP image evaluation. The results showed that the peak signal-to-noise ratio (PSNR) and feature similarity (FSIM) of the AD-CNNnet method were significantly higher than those of traditional methods, while the normalized mean square error (NMSE) was significantly lower than that of traditional algorithms (*P* < 0.05). 80 cases were positive by CTP-CTA, including 16 cases of hyperacute ischemic stroke and 64 cases of acute ischemic stroke. The diagnostic sensitivity was 93.66%, and the specificity was 96.18%. The cerebral blood flow (CBF), cerebral blood volume (CBV), and the mean transit time (MTT) in the infarcted area were significantly greater than those in the corresponding healthy side area, and the time to peak (TTP) was significantly less than that in the corresponding healthy side area (*P* < 0.05). The cerebral perfusion parameters CBF, TTP, and MTT in the penumbra were significantly different from those in the infarct central area and the corresponding contralateral area, and TTP was the most sensitive (*P* < 0.05). To sum up, deep learning algorithm-based CTP combined with CTA could find the location of cerebral infarction lesions as early as possible to provide a reliable diagnostic result for the diagnosis of ultra-early acute ischemic stroke.

## 1. Introduction

Ischemic stroke is the most common type of stroke, accounting for about 80% of all strokes. It is the softening and necrosis of brain tissue caused by blood circulation disorder, ischemia, and hypoxia in the local brain tissue, namely, vascular blockage [1–3]. The symptoms of acute ischemic stroke are mainly sudden skewing of the mouth and eyes with saliva secretion. Patients will not only have unclear speech but also have difficulty in pronunciation. In addition, some patients will have aphasia, dysphagia, weakness, or numbness of one limb [4]. At present, it is generally believed that the main factors causing acute ischemic stroke include large atherosclerosis, cardiogenic embolism, and arteriolar occlusion [5]. The inducing factors included age, race, heredity, hypertension, diabetes, dyslipidemia, heart disease, mental state, and so on [6, 7]. Acute ischemic stroke has the characteristics of high incidence rate, high mortality rate, high disability rate, and high recurrence rate. According to statistics, about one person dies of stroke every six seconds, and one person may be disabled by stroke every six seconds [8]. Therefore, early detection of the existence of early ischemic penumbra and diagnosis of acute ischemic stroke are very critical for the therapeutic effectiveness and prognosis of patients.

Imaging is used in the clinical diagnosis of acute ischemic stroke. Plain CT scan is the first choice for screening suspected stroke, which can distinguish intracranial hemorrhage and nonvascular lesions. However, it is difficult to find and diagnose the disease early. Generally, it cannot be found until 24 hours after ischemia [9–11]. Conventional MRI is effective in displaying acute small infarct and posterior circulation ischemic stroke. At present, the mismatch between PWI and DWI of MRI is a more effective method to judge the ischemic penumbra, but MRI has some limitations, such as long examination time, many contraindications, and high examination cost [12, 13]. CT perfusion imaging is a common method to evaluate acute ischemic stroke at present. It can early display the focus of cerebral ischemia and distinguish the inactivated brain tissue and ischemic penumbra. It has important clinical significance for timely diagnosis and guiding treatment [14]. CT angiography (CTA) is mainly through intravenous injection of drugs. When the drugs pass through the vascular arteries, they are scanned by CT. The formed images are imaged by computer synthesis. CTA can display the blocking site, vascular size, and blood flow compensation of patients with acute ischemic stroke [15]. Therefore, this study intends to use CT perfusion (CTP) imaging and CTA in the diagnosis of acute ischemic stroke.

Deep learning is a branch of machine learning. It is an algorithm that attempts to abstract data at a high level using multiple processing layers composed of complex structures or multiple nonlinear transformations. So far, several deep learning frameworks have been applied in the fields of computer vision, speech recognition, natural language processing, medicine, and bioinformatics [16].

Convolutional neural network (CNN) could share convolution kernels and process high-dimensional data without pressure. CNN enabled the image to still retain the original position relationship through convolutional operation with good image processing effects. However, it showed some disadvantages, including the high demand for sample size and strong hardware dependence. In summary, 88 patients with acute ischemic stroke were examined with CTP and CTA images, and the deep learning algorithm was applied to the original image processing. The diagnostic sensitivity, specificity, and cerebral perfusion parameters were analyzed to confirm the application value of CTP imaging based on a deep learning algorithm combined with head and neck CTA in the diagnosis of ultra-early acute ischemic stroke, which provided help for the clinical diagnosis and treatment of acute ischemic stroke.

## 2. Materials and Methods

### 2.1. Research Object

Eighty-eight patients with acute ischemic stroke in the hospital from May 2019 to May 2021 were collected as the research objects, including 54 males and 34 females, aged 33–79 years. According to this study, it was approved by the medical ethics committee of the hospital. The patients and their families understood the study and signed the informed consent.

Inclusion criteria: (1) patients diagnosed with acute ischemic stroke due to numbness, hemiplegia, weakness of one limb, and aphasia; (2) the time from symptom onset to baseline imaging examination was within 24 hours; (3) cranial CT excluded intracerebral hemorrhage; (4) complete clinical data; and (5) the National Institutes of Health Stroke Scale (NIHSS) score was greater than four.

Exclusion criteria: (1) complicated with mental diseases; (2) poor inspection compliance; (3) allergic constitution; and (4) patients who withdrew from the experiment halfway.

### 2.2. Inspection Method

CTP: after the cerebral hemorrhage was excluded by a routine CT plain scan, CTP imaging was performed. 42 mL of contrast agent iodopropane and 20 mL normal saline were injected through elbow vein at the rate of 6 ml/s. The scanning range was parietal bone, 15 cm. The time density curve was obtained. After image processing, the cerebral blood flow (CBF), cerebral blood volume (CBV), mean transit time (MTT), and time to peak (TTP) were obtained. The parameters such as CBF, CBV, TTP, and MTT in the corresponding areas of the affected side and the healthy side were measured by mirror technique, and the perfusion parameters in the lesion area (infarct core and penumbra) and the corresponding healthy side were compared.

CTA: scanning range was aortic arch cranial apex. 55 mL iopromide reagent was injected through the median elbow vein at the injection rate of 4.5–5.0 mL/s, and then 55 mL normal saline was injected. Scanning parameters: voltage 120 kV, current 240 mA, and layer thickness 0.45 mm. According to the location of the lesion, it was divided into: infratentorial lesion, paraventricular and basal ganglia lesions, frontoparietal lobe lesions, temporal occipital lobe lesions, and the lesions involving a large area of one cerebral hemisphere. The infarct volume was calculated.

### 2.3. Computed Tomography Perfusion Deconvolution Algorithm on Deep Learning

In CTP image processing, if the contrast agent concentration at the pulse input was *D*_*ca*_, the region of interest was *V*_*RI*_, and the corresponding average time density curve was *TDC*_*RI*_; the relationship between *D*_*ca*_ and *TDC*_*RI*_ could be expressed as follows:

(1) $$\begin{array}{c} TDC_{RI}\left(t\right)=\left(D_{ca}\times U\right)\left(t\right). \end{array}$$

In the above equation, *U*(*t*) represents the residual function of blood flow scale. The above equation could be solved by deconvolution. In numerical implementation, the convolution equation (1) could be expressed by matrix multiplication after discretization. The volume of interest containing N voxels was taken as an example.

(2) $$\begin{array}{c} \overset{⌢}{U}=\arg_{U}^{\min\left({\left\|NU-D\right\|}_{2}^{2}+\alpha E\left(U\right)/2\right)}. \end{array}$$

In the above equation, *N* represents a block cyclic matrix, $N\in E^{\tilde{K}\cdot \tilde{K}}$ and *K* represent dynamic scanning parameters, (‖*NU* − *D*‖_2_^2^/2) represent fidelity terms, *E*(*U*) represent regular terms, and *α* represent weight parameters.

To solve (1), an auxiliary variable *Z* was introduced into the blood flow scale residual function and the alternating direction multiplier method (ADMM) [17] was used, and the process could be expressed as follows:

(3) $$\begin{array}{c} U^{\left(n\right)}=\left(1-b_{su}\chi \right)U^{\left(n-1\right)}+b_{su}\chi \left(Z^{\left(n-1\right)}-\lambda^{\left(n-1\right)}\right)-b_{su}N^{\tau }\left(NU^{\left(n-1\right)}-D\right),\\ Z^{\left(n\right)}=\left(1-b_{su}\chi \right)Z^{\left(n-1\right)}+b_{sz}\chi \left(U^{\left(n\right)}+\lambda^{\left(n-1\right)}\right)-\alpha \Lambda E\left(Z^{\left(n-1\right)}\right),\\ \lambda^{\left(n\right)}=\lambda^{\left(n-1\right)}+\kappa \left(U^{\left(n\right)}-Z^{\left(n\right)}\right). \end{array}$$

In the above equations, *λ* represents a scaled Lagrange multiplier, *χ* represents a penalty hyperparameter, *τ* represents a transpose operator, *b*_*su*_ represents a step size *U*^(*n*)^, *b*_*sz*_ represents a step size *Z*^(*n*)^, Λ represents a regular term gradient operator, and *κ* represents a learning rate.

For the modular structure of ADMM algorithm, the regular term of (2) was separated from deconvolution. For example, *U*^(*n*)^ was deconvolution process, *Z*^(*n*)^ was denoising process, and *λ*^(*n*)^ was iterative update auxiliary variable. Then, based on the idea of plug and play, the deconvolution process of low-dose CTP was constrained. The equations were improved as follows:

(4) $$\begin{array}{c} U^{\left(n\right)}=\left(1-{\tilde{\chi }}^{\left(n\right)}\right)U^{\left(n-1\right)}+{\tilde{\chi }}^{\left(n\right)}\left(Z^{\left(n-1\right)}-\lambda^{\left(n-1\right)}\right)-{\tilde{b}}_{su}^{\left(n\right)}N^{\tau }\left(NU^{\left(n-1\right)}-D\right),\\ Z^{\left(n\right)}=\left(1-{\tilde{\chi }}^{\left(n\right)}\right)Z^{\left(n-1\right)}+{\tilde{\chi }}^{\left(n\right)}\left(U^{\left(n\right)}+\lambda^{\left(n-1\right)}\right)-\tilde{\alpha }{\text{Res}}^{\left(n,l\right)}\left(Z^{\left(n-1\right)}\right),\\ \lambda^{\left(n\right)}=\lambda^{\left(n-1\right)}+\kappa^{\left(n\right)}\left(U^{\left(n\right)}-Z^{\left(n\right)}\right),\\ \tilde{\chi }=b_{su}\chi . \end{array}$$

Compared with before, the update step size and penalty super parameters were combined into one parameter, and the performance of deconvolution network model could be improved by adaptively adjusting the parameters. The operation process of the deep learning deconvolution network model designed in this paper could be set as AD-CNNnet (Figure 1).

### 2.4. Simulation Experiment

The experiment was conducted on the platform of MATLAB 2015b.  Table 1 revealed the parameter settings.

Block cyclic truncated singular value decomposition (bSVD) [18], sparse perfusion deconvolution (SPD) [19], and DenseSRNet [20] were used as comparison methods with AD-CNNnet.

Peak signal-to-noise ratio (PSNR), normalized mean square error (NMSE), and feature similarity (FSIM) were selected as evaluation indexes [21].

### 2.5. Statistical Methods

The data of this study were analyzed by SPSS19.0 statistical software. The measurement data were expressed by mean ± standard deviation (‾*x* ± *s*), and the counting data were expressed by percentage (%). One-way analysis of variance was used for pairwise comparison. The difference was statistically significant (*P* < 0.05).

## 3. Results

### 3.1. Performance Analysis Results of Network Model

Firstly, the optimal values of three parameters: the number of model filters, the number of residual blocks, and the number of ADMM iteration steps, were analyzed to live the best deconvolution network model for image processing.

If the number of filters was set to 5, 10, and 15, the loss curve of the model in network training could be illustrated in Figure 2. The loss curve under the three filter parameters decreased rapidly with the enhancement of network training times until it tended to be stable. Among them, the model with 15 filters has the best loss curve and the more stable learning ability.

If the number of residuals was set to 3, 5, and 7, the loss curve of the model in network training could be expressed in Figure 3. The loss curve under the three residual parameters decreased rapidly with the increase of network training times until it tended to be stable. Among them, the model with 7 residuals had the best loss curve and more stable learning ability.

If the number of ADMM iteration steps was set to 6, 9, and 12, the loss curve of the model in network training could be illustrated in Figure 4. The loss curve under the three iteration steps decreased rapidly with the increase of network training times until it tended to be stable. Among them, the model loss curve with 12 iterative steps of ADMM was the best and had more stable learning ability.

In terms of visual evaluation (Figure 5), the perfusion parameter map obtained by bSVD method was damaged by noise induced artifacts. The perfusion parameter map obtained by SPD and DenseSRNet methods was too smooth. The perfusion parameter map obtained by AD-CNNnet method performed best in suppressing artifacts and preserving details, which was closer to the reference image.

In terms of quantitative evaluation (Figure 6), PSNR and FSIM of AD-CNNnet method were significantly higher than those of other methods, while NMSE was significantly lower than other algorithms, and the difference was statistically significant (*P* < 0.05).

### 3.2. Computed Tomography Perfusion-Computed Tomography Angiography Inspection Results

Figure 7 shows that among the 88 patients, CTP-CTA was negative in 8 cases, including 2 cases of pons, 1 case of lacunar infarction in the left basal ganglia, 2 cases of multiple punctate acute cerebral infarction in the right frontal parietal lobe, and 3 cases of transient ischemic attack. CTP-CTA was positive in 80 cases, including 16 cases of hyperacute ischemic stroke and 64 cases of acute ischemic stroke. The diagnostic sensitivity was 93.66%, and the specificity was 96.18%.

### 3.3. Comparison of Cerebral Perfusion Parameters between Infarcted Area and Contralateral Area

Figure 8 reveals that the cerebral perfusion parameters CBF, CBV, and MTT in the infarcted area were significantly greater than those in the corresponding contralateral area, and the difference was statistically significant (*P* < 0.05). The cerebral perfusion parameter TTP in the infarcted area was significantly lower than that in the corresponding contralateral area, and the difference was statistically significant (*P* < 0.05).

### 3.4. Comparison of Cerebral Perfusion Parameters in Penumbra, Infarct Center, and Contralateral Area

Figure 9 indicates that the cerebral perfusion parameters CBF, TTP, and MTT in the penumbra were significantly different from those in the infarct central area and the corresponding healthy side area (*P* < 0.05). The cerebral perfusion parameter CBV in the penumbra was significantly different from that in the infarct center (*P* < 0.05), but not from the corresponding healthy side (*P* > 0.05).

### 3.5. Analysis of Case Data of Some Patients

CTA indicated that the left anterior cerebral artery of male, 58, was thin (Figure 10), the distal end was not developed, and the P2 segment of the left posterior cerebral artery was blocked. CTP showed that CBV, CBF, and MTT decreased in the core area of cerebral infarction. TTP prolonged significantly. The volume of hypoperfusion area was 18.7 mL, and the penumbra was large.

CTA revealed the occlusion of the intracranial segment of the right internal carotid artery and the right middle cerebral artery of a female, 65 (Figure 11). CTP showed that CBV, CBF, and MTT decreased in the core area of cerebral infarction, and TTP prolonged significantly.

## 4. Discussion

Cerebral infarction was the main cause of disability at present. Timely and rapid recovery of cerebral blood flow in patients with acute cerebral infarction has become an effective way to reduce the disability rate. Clinically, it was found that strict time limit can improve the effect of intravenous thrombolytic therapy by about 10%. Therefore, the limited time window has certain limitations. Rapid and accurate judgment of ischemic penumbra has become the key to the treatment of cerebral infarction [22]. In this study, 88 patients with acute ischemic stroke in the hospital were selected as the research object, and the brain CTP and CTA were examined by SOMATOM spirit double-slice spiral CT. To improve the effect of image diagnosis, a new deconvolution network model AD-CNNnet based on deep learning was proposed and used in actual CTP image evaluation. Firstly, the application effect of the model was analyzed. It was found that the perfusion parameter map obtained by AD-CNNnet method performs best in suppressing artifacts and preserving details, which was closer to the reference image, and has the best effect compared with other methods. In terms of quantitative evaluation, PSNR and FSIM of AD-CNNnet method were significantly higher than those of other methods, while NMSE was significantly lower than other algorithms (*P* < 0.05). PSNR and NMSE were two widely used objective image quality indicators. The larger the PSNR was, the smaller the NMSE was, and the better the image quality was. FSIM was used to measure the perceived similarity of two images. The closer the value was to 1, the higher the image similarity was proved [23]. The results gave that the proposed AD-CNNnet model showed more significant robustness in parameter calculation and could improve imaging quality more obviously compared with traditional algorithms.

CTP and CTA based on AD-CNNnet model were applied to the diagnosis of 88 patients with acute ischemia. It was found that 80 patients were positive for CTP-CTA, including 16 cases of hyperacute ischemic stroke and 64 cases of acute ischemic stroke. The diagnostic sensitivity was 93.66% and the specificity was 96.18%, which was similar to the results of Hakim A et al. (2019) [24]. Previous studies [25] showed that the low-density lesions could only be displayed by routine CT in patients with cerebral ischemia 24 hours after onset. In the early stage of acute cerebral infarction, especially in the hyperacute stage <6 h, the sensitivity and diagnostic rate of conventional CT plain scan were very low, indicating that CTP-CTA based on deep learning algorithm could find the location of cerebral infarction lesions as soon as possible. It provided a reliable clinical basis for the diagnosis of ultra early cerebral infarction and had a high clinical application value. By comparing the cerebral perfusion parameters in different regions, it was found that the CBF, CBV, and MTT in the infarcted area were significantly higher than those in the corresponding healthy side area. Besides, the TTP was significantly lower than that in the corresponding healthy side area. The difference was statistically significant (*P* < 0.05), indicating that the cerebral perfusion parameters CBF, CBV, MTT, and TTP can predict the occurrence of acute cerebral infarction to a certain extent [26]. Further analysis showed that the cerebral perfusion parameters CBF, TTP, and MTT in the penumbra were significantly different from the infarct central area and the corresponding contralateral area. TTP was the most sensitive (*P* < 0.05), which showed that the cerebral perfusion parameters CBF, TTP, and MTT had a good indicating significance for evaluating the penumbra area.

## 5. Conclusion

In this study, 88 patients with acute ischemic stroke in the hospital were taken as the research object, and the brain CTP and CTA were examined by SOMATOM Spirit double-slice spiral CT. To improve the effect of image diagnosis, a new deconvolution network model AD-CNNnet based on deep learning was proposed and used in patient CTP image evaluation. The results showed that CTP-CTA based on AD-CNNnet model could find the location of cerebral infarction as soon as possible, which provided a reliable clinical basis for the diagnosis of ultra early cerebral infarction and had a high clinical application value. In addition, its cerebral perfusion parameters CBF, CBV, MTT, and TTP can assist in judging the ischemic penumbra to a certain extent and provide guidance for individualized treatment of patients. However, there were few patients selected in this study and the source was single, which may have some impact on the results. In addition, the long-term follow-up data of patients were not collected, and the image evaluation of patient prognosis was not involved. More patient sample data will be collected in the later study to further explore the application value of CTP combined with CTA based on deep learning algorithm in the prognosis of patients with acute ischemic stroke. In conclusion, the results of this study provide a reference for the combined application of artificial intelligence technology and clinical imaging.

## Figures and Tables

**Figure 1:** Improved deep learning deconvolution network model.

**Figure 2:** Loss curve of model training under different filter numbers.

**Figure 3:** Loss curve of model training under different number of residual blocks.

**Figure 4:** Loss curve of model training under different ADMM iteration steps.

**Figure 5:** Perfusion parameters obtained by deconvolution network model. A was the reference image; B was SPD; C was bSVD; D was DenseSRNet; E was AD-CNNnet.

**Figure 6:** Quantitative evaluation indicators of deconvolution network model. (a) PSNR; (b) NMSE; (c) FSIM. *∗* indicates that the difference between AD-CNNnet and other methods was statistically significant (*P* < 0.05).

**Figure 7:** CTP-CTA results.

**Figure 8:** Comparison of cerebral perfusion parameters between infarcted area and contralateral area. A represents CBF and CBV; B represents MTT and TTP. *∗* indicates that there was significant difference between infarcted area and healthy side area (*P* < 0.05).

**Figure 9:** Comparison of cerebral perfusion parameters in penumbra, infarct center, and contralateral area of patients. A refers to CBF and CBV; B refers to MTT and TTP. *∗* indicates that the difference between the penumbra area, the infarcted area, and the contralateral area was statistically significant (*P* < 0.05).

**Figure 10:** A 58-year-old male patient with left limb weakness and unclear speech was admitted to the hospital for 8 hours. A was CTA image; B was CTP image; and C-F was CBV, CBF, MTT, and TTP perfusion images, respectively.

**Figure 11:** A 65-year-old male patient with sudden weakness of left upper limb and unclear consciousness was admitted to the hospital for 5 hours. A was CTA image; B was CTP image; C-F was CBV, CBF, MTT, and TTP perfusion images, respectively.

**Table 1:** Network model parameter setting.

Parameter	Numerical value
Number of network residual blocks	7
Number of network filters	15
Filter size	3 × 3
ADMM iteration steps	12
Initial learning rate	4500

## Data Availability

The data used to support the findings of this study are available from the corresponding author upon request.
